This article has been retracted.

# To Explore the Effects of Acupuncture and Medical Treatment at Different Times on the Gastrointestinal Reaction and White Blood Cell Count of Patients with Lung Cancer Chemotherapy

**DOI:** 10.1155/2022/5261344

**Published:** 2022-04-07

**Authors:** Qingchun Zhao, Hui Du, Jinghao Liu, Yu Hua, Xiaoyu Niu, Jun Chen

**Affiliations:** Department of Lung Cancer Surgery, Tianjin Medical University General Hospital, Tianjin, China

## Abstract

**Objective:**

To explore and analyze the effects of acupuncture and medical treatment at different times on the gastrointestinal reaction and leukocyte count of patients with lung cancer undergoing chemotherapy.

**Methods:**

Select 224 lung cancer chemotherapy patients admitted to our hospital and randomly divide them into three groups: control group (*n* = 76), study 1 group (*n* = 78), and study 2 group (*n* = 70). The control group was treated with tropisetron hydrochloride for 30 minutes before chemotherapy. Study 1 group was given tropisetron hydrochloride and acupuncture combination therapy 30 minutes before chemotherapy. Study 2 group was given tropisetron hydrochloride treatment 30 min before chemotherapy and acupuncture treatment 30 min after chemotherapy. Collect patients' general information and compare the three groups of white blood cell count, G-CSF, GM-CSF levels, quality of life and KPS score, platelets, neutrophils, hemoglobin levels, TCM symptom scores, and the degree of digestive tract reaction.

**Results:**

The data of the control group and study groups 1 and 2 are comparable in gender, age, pathological type, etc. (*P* > 0.05). Before treatment, the white blood cell counts of the three groups were not significantly different (*P* > 0.05), significantly reduced after treatment, but the difference between the groups was not statistically significant (*P* > 0.05). The levels of G-CSF and GM-CSF in the three groups were not substantially different before treatment (*P* > 0.05). The levels of G-CSF and GM-CSF were considerably lowered in all three groups, although the drop in the study group was more significant (*P* > 0.05) when compared to that in the control group. Before treatment, the quality of life and KPS score of the three groups were not statistically different (*P* > 0.05). The three groups' quality of life and KPS scores fell after treatment, with the study 1 group experiencing the greatest reduction, followed by the study 2 group and the control group. The levels of platelets, neutrophils, and hemoglobin in all three groups declined dramatically, with the most noticeable reduction in the control group, followed by study 2 and study 1. The difference between the three groups was statistically significant (*P* < 0.05). The TCM symptom scores of the three groups showed an upward trend, but compared with those of the study 1 group and study 2 group, the TCM symptom scores of the control group increased significantly and the difference between the three groups was statistically significant (*P* < 0.05). The effective rates of the control group, study group 1, and study group 2 were 42.11%, 82.05%, and 62.86%, respectively; compared with that of the control group, the treatment efficiency of study groups 1 and 2 was higher and the difference between the three groups was statistically significant (*P* < 0.05).

**Conclusion:**

Tropisetron hydrochloride is an effective treatment for patients with lung cancer before chemotherapy, which can effectively improve the side effects of nausea and vomiting caused by chemotherapy, reduce the white blood cell count, and improve the quality of life of patients; it plays an important role in the improvement of prognosis.

## 1. Introduction

Lung cancer is a primary lung tumor with a high incidence rate among middle-aged persons and the maximum death rate in my nation; clinical data suggest that the prevalence of this illness is climbing year by year [1]. Non-small cell lung cancer and small cell lung cancer are the two most frequent types of lung cancer. Chemotherapy seems to be the most common treatment for this condition. Chemotherapy may cause nausea and vomiting, among other adverse effects [2]. Severe vomiting may result in dehydration, electrolyte imbalances, and malnutrition, lowering resistance and jeopardizing the patient's relatively normal life. Negative emotions are severe, and they affect the therapeutic impact directly [3, 4]. Despite the fact that traditional chemotherapy has a reasonable effect, the patient has nausea and vomiting, which is detrimental to the patient's prognosis, and the patient's compliance is insufficient. Nondrug treatment should be used to prevent gastrointestinal effects. Negative emotions are severe, and they will have a significant impact on the therapy effect [3, 4]. Although traditional chemotherapy has a satisfactory effect, the patient experiences nausea and vomiting, which is detrimental to the patient's prognosis, and the patient's compliance is low. To avoid gastrointestinal problems, nondrug treatment should be employed. Some scholars pointed out [5] that the effect of acupuncture treatment on lung cancer patients undergoing chemotherapy is significant. The study selected 224 patients undergoing chemotherapy for lung cancer in our hospital. The patients were treated with acupuncture and tropisetron hydrochloride to analyze the safety of the treatment and its effect on the white blood cell count. The relevant content is now reported as follows.

## 2. Materials and Methods

### 2.1. Data

Select 224 lung cancer chemotherapy patients admitted to our hospital and randomly divide them into 3 groups: control group (*n* = 76), study 1 group (*n* = 78), and study 2 group (*n* = 70). The control group (*n* = 76) has 43 males and 33 females, aged 38–86 years (average age 35.76 ± 2.42 years). The study 1 group (*n* = 78) has 46 males and 32 females, aged 38–85 (average age 35.62 ± 2.31 years). The study 3 group (*n* = 70) has 38 males and 32 females, aged from 38 to 85 (average age 35.45 ± 2.24 years). The subjects agreed with the study, the data were comparable (*P* > 0.05), and the hospital ethics committee agreed.

Inclusion criteria [6] are as follows: (1) Karnofsky score above 60 points, (2) expected survival cycle > 6 months, (3) normal, (4) can accept prognostic follow-up, (5) normal cognitive function and cooperative with the study, (6) normal coagulation and liver and kidney function, and (7) meet the diagnostic criteria for lung cancer. After diagnosis, he was diagnosed with lung cancer.

Exclusion criteria are as follow: (1) allergy to study drugs; (2) intolerance to acupuncture; (3) patients during pregnancy or lactation; (4) central nervous system disorders; (5) patients with hyperuricemia, chickenpox, or gout; and (6) Parkinson's syndrome.

### 2.2. Methods

In the control group, 30 ml of tropisetron hydrochloride (National Medicine Zhunzi H20050535, Qilu Pharmaceutical Co. Ltd.) was given 30 minutes before chemotherapy, dissolved in 0.9% saline, intravenously injected at a rate of 60 ml/h, and finished within 30 minutes. Patients were treated once a day for 5 consecutive days.

Tropisetron hydrochloride and acupuncture combination treatment were administered 30 minutes before chemotherapy at Neiguan, Zusanli, and Zhongwan acupuncture sites.

Tropisetron hydrochloride was administered 30 minutes before chemotherapy, and acupuncture was given 30 minutes after chemotherapy in study group 2. The procedure is as follows: the patient is positioned in a supine posture, the skin is sterilized locally, Neiguan, Zusanli, and Zhongwan are chosen, and 1.5 inch needles are used. Puncture 0.5–1 cun straight at Neiguan, take the flexor carpi radialis tendon and palmar longus tendon, and puncture 2 cun above the transverse crease of the wrist; stab Zusanli 1.0–1.5 cun straight and take 1 horizontal finger outside the anterior tibial crest, Dubi point 3 cun below; pierce 1.0–1.5 cun straight into the middle cavity, 4 cun above the umbilicus, on the anterior midline. After getting Qi by acupuncture at Neiguan, Zusanli, and Zhongwan acupoints, the needles were kept for half an hour. During this period, the needles were given once every 10 minutes, once a day, for a total of 5 days of continuous treatment.

### 2.3. Outcome Measurement

#### 2.3.1. Three Sets of General Data Analysis

The gender, age, pathological type (adenosquamous carcinoma, small cell lung cancer, large cell lung cancer, squamous cell carcinoma, and adenocarcinoma), etc. are included.

### 2.4. Comparison of Three Groups of White Blood Cell Counts [7]

Use an automatic blood cell analyzer to detect the level of white blood cells, and the relevant operations are carried out in accordance with the instructions.

### 2.5. Comparison of G-CSF and GM-CSF Levels in the Three Groups [8]

3 ml of fasting venous blood was drawn, centrifuged at 3500 rpm for 10 minutes, and the serum was obtained and detected by an automatic blood cell analyzer.

### 2.6. Compare the Life Quality of the Three Groups and KPS Score [9]

The quality of life was assessed using the SF-36 scale, which has a total score of 100. Patients' functional state is assessed using the Karnofsky functional status scoring system. A total of 100 points is awarded. The smaller the frequency of adverse responses and the better the health state, the higher the score.

### 2.7. Compare the Levels of Platelets, Neutrophils, and Hemoglobin in the Three Groups [10]

The levels of platelets, neutrophils, and hemoglobin should be detected by an automatic blood cell analyzer.

### 2.8. Comparison of the Three Groups of TCM Symptom Scores

Poor complexion, fatigue, poor appetite, shortness of breath, and spontaneous sweating are included.

### 2.9. Comparison of Digestive Tract Reaction Degree after Three Groups of Chemotherapy [11]

Grades III and IV indicate ineffectiveness, and there is no significant improvement or increase in the length of the lesion; grade II indicates mild remission; grade I indicates partial effect; grade 0 indicates complete effect; the effective rate is (II + I + 0) number of cases/the total number of cases, multiplied by 100%.

### 2.10. Statistical Methods

Enter the acquired data into the EXCEL form, analyze the data using the statistical SPSS22.0 program, and perform a normal distribution test on the data. If the data are normal, the composition ratio and rate, as well as the difference between the groups' compositions, should be used to explain the count data. For sex analysis, the chi-square test is used, measurement data is reported as mean standard deviation, the *t*-test is used to compare groups, the physical influencing elements of the case group are analyzed using logistic regression, and *P* < 0.05 is regarded statistically significant. GraphPad Prism 8 is the graph program utilized by the institution.

## 3. Results

### 3.1. Three Sets of General Data Analysis

The data of the control group, study 1 group, and study 2 group, such as gender, age, and pathological type, are comparable (*P* > 0.05, Table 1).

### 3.2. Comparison of Three Groups of White Blood Cell Counts

Before treatment, there was no significant difference in white blood cell count between the three groups (*P* > 0.05). After treatment, the white blood cell counts of the three groups were significantly reduced, but the difference between the groups was not statistically significant (*P* > 0.05, Table 2).

### 3.3. Comparison of G-CSF and GM-CSF Levels in the Three Groups

The levels of G-CSF and GM-CSF in the three groups did not vary significantly before treatment (*P* > 0.05). The levels of G-CSF and GM-CSF in all three groups were considerably lowered after treatment; however, the drop in the study group was more significant (*P* < 0.05) when compared to that in the control group (see Table 3).

Before treatment, there was no significant difference in the quality of life and KPS score between the three groups (*P* > 0.05). After treatment, the quality of life and KPS scores of the three groups decreased. The decrease was the most obvious in the study 1 group, followed by study 2 and the control group. ^#^ indicates that the difference between the three groups was statistically significant (*P* < 0.05), as shown in Figure 1.

The levels of platelets, neutrophils, and hemoglobin in the three groups were not significantly different before therapy (*P* > 0.05). Platelets, neutrophils, and hemoglobin levels in all three groups declined considerably after treatment, with the control group showing the greatest reduction, followed by study 2 and study 1. As illustrated in Figure 2, ^#^ indicates that the difference between the three groups is statistically significant (*P* < 0.05).

Before treatment, there was no significant difference in the scores of clinical symptoms such as poor complexion, fatigue, poor appetite, shortness of breath, and spontaneous sweating among the three groups. After treatment, the scores of TCM symptoms in the three groups showed an upward trend, but compared with study 1 and study 2, the TCM symptom score of the control group increased significantly and the difference between the three groups was statistically significant (*P* < 0.05), as shown in Figure 3.

The effective rates of the control group, study group 1, and study group 2 were 42.11%, 82.05%, and 62.86%, respectively. Compared with that of the control group, the treatment efficiency of study groups 1 and 2 was higher. Compared with those of the three groups, the difference was statistically significant. Significance was *P* < 0.05, as shown in Figure 4.

## 4. Discussion

Nausea and vomiting occur in the stomach, which is classified as “fullness” and “vomiting.” Gastrointestinal responses are caused by a variety of reasons, including weak internal organs, six external kinks, psychiatric problems, and medication toxicity [12, 13]. Chemotherapy would harm the natural tissues of the spleen and stomach, resulting in an imbalance of bodily fluid infusion, buildup of phlegm in the liver, the general etiology of gastric failure, and decrease of qi, according to TCM oncology. Drugs are the primary source of unpleasant responses including chemotherapy-induced vomiting, according to experts. If a patient suffers from despair, anxiety, or other negative feelings, the spleen and stomach will be severely damaged, affecting their function, and nausea and vomiting will be exacerbated [14–16]. Acupuncture and moxibustion therapy on patients have the effect of regulating qi and blood, channeling meridians, and improving yin and yang balance, as well as efficiently preventing and treating diseases [17]. The gastrointestinal response produced by chemotherapy may be eliminated with acupuncture at Neiguan, Zusanli, and Zhongwan; the KPS score is greatly enhanced, and the therapeutic impact of acupuncture coupled with medications is more visible [18, 19].

The results of the study showed that the effective rates of the control group, study group 1, and study group 2 were 42.11%, 82.05%, and 62.86%, respectively. Compared with the control group, study groups 1 and 2 had higher effective treatment rates. Comparing the results of the three groups. The difference was statistically significant (*P* < 0.05). The results confirmed that acupuncture at Neiguan, Zusanli, Zhongwan, etc. can improve the body's condition and adjust its functions to avoid external stimuli from damaging the body. In addition, the results of the study showed that the quality of life and KPS scores in the three groups decreased. The decrease in study group 1 was the most obvious, followed by study group 2 and the control group. The difference between the three groups was statistically significant (*P* < 0.05). The results confirmed that compared with the treatment of tropisetron hydrochloride alone, the combined acupuncture treatment can improve the life quality of the patients to a greater extent, which is beneficial to the improvement of the patient's physical function status, and the patient's self-confidence in treatment is significantly improved. The patient was treated with chemotherapy, and the side effects and white blood cell count decreased significantly [20–22]. The results of combined acupuncture and drug treatment showed that the white blood cell counts of the three groups were significantly reduced after treatment, but the difference between the groups was not statistically significant (*P* > 0.05). The results confirmed that acupuncture will affect the white blood cell count to a large extent but the difference is not obvious, which may be related to the main purpose of acupuncture and the treatment time, so we should explore this aspect in more depth.

This research looked at the effects of acupuncture and medication treatment on platelets, neutrophils, and hemoglobin levels in lung cancer patients who were receiving chemotherapy. The research's findings revealed that platelets, neutrophils, and hemoglobin levels in all three groups declined considerably, with the largest reduction in the control group, followed by study 2 and study 1. There was a statistically significant difference between the three groups (*P* < 0.05). Acupuncture and medication treatment may significantly lower platelets, neutrophils, and hemoglobin levels, according to the findings, although treatment 30 minutes before chemotherapy has a more noticeable impact. The therapy technique may increase the levels of G-CSF and GM-CSF while also slowing the advancement of the illness and reducing patients' clinical symptoms. It should also be mentioned that while treating patients in a professional setting, the amount of time spent on acupuncture should be tightly limited [23, 24]. The clinical symptoms of patients with lung cancer are obvious. The results of the study show that the TCM symptom scores of the three groups are on the rise, but compared with those of the study 1 group and the study 2 group, the TCM symptom scores of the control group have increased significantly and the difference between the three groups is statistically significant (*P* < 0.05). The results confirmed that compared with drug therapy alone, combined acupuncture treatment can relieve clinical symptoms to a greater extent and the effect of tropisetron hydrochloride administered 30 minutes before chemotherapy and acupuncture treatment 30 minutes after chemotherapy is more significant.

In summary, tropisetron hydrochloride treatment for lung cancer patients undergoing chemotherapy before chemotherapy has ideal results. It can effectively improve the adverse reactions of nausea and vomiting caused by chemotherapy, reduce white blood cell counts, and improve the life quality of patients. The improvement of prognosis plays a very important role.

## Figures and Tables

**Figure 1:** Compare the life's quality and KPS scores of the three groups.

**Figure 2:** Compare the levels of platelets, neutrophils, and hemoglobin in the three groups.

**Figure 3:** Compare the scores of the three groups of TCM symptoms.

**Figure 4:** Comparison of digestive tract reaction degree after three groups of chemotherapy.

**Table 1:** Three sets of general data analysis.

Group	Number of cases	Gender		Age	Pathological type				
		Male	Female		Adenosquamous carcinoma	Small cell lung cancer	Large cell lung cancer	Squamous cell carcinoma	Adenocarcinoma
Control group	76	43 (56.58)	33 (43.42)	35.76 ± 2.42	2 (2.63)	16 (21.05)	2 (2.63)	18 (23.68)	38 (50.00)
Study group 1	78	46 (58.97)	32 (41.03)	35.62 ± 2.31	4 (5.13)	12 (15.38)	2 (2.56)	14 (17.95)	46 (58.97)
Study group 2	70	38 (54.29)	32 (45.71	35.45 ± 2.24	2 (2.86)	10 (14.29)	4 (5.71)	20 (28.57)	34 (48.57)

**Table 2:** Comparison of three groups of white blood cell counts ($\bar{x}\pm s$).

Group	Number of cases	Before therapy	After treatment	Difference
Control group	76	5.56 ± 0.99	4.25 ± 0.62	1.31 ± 0.37
Study group 1	78	5.61 ± 0.92	4.68 ± 0.79	0.93 ± 0.13
Study group 2	70	5.65 ± 0.96	4.48 ± 0.72	1.17 ± 0.24
*F*	/	1.524	1.365	1.472
*P*	/	>0.05	>0.05	>0.05

**Table 3:** Comparison of G-CSF and GM-CSF levels in the three groups ($\bar{x}\pm s$).

Group	Number of cases	G-CSF (ng/L)		GM-CSF (ng/L)	
		Before therapy	After treatment	Before therapy	After treatment
Control group	76	406.92 ± 49.05	281.11 ± 30.42	31.05 ± 7.65	25.59 ± 5.94
Study group 1	78	406.64 ± 48.57	246.32 ± 24.39	30.53 ± 7.81	23.57 ± 5.05
Study group 2	70	403.51 ± 48.38	223.53 ± 23.18	30.40 ± 7.73	21.94 ± 4.29
*F*	/	1.635	18.254	0.421	16.724
*P*	/	>0.05	<0.05	>0.05	<0.05

## Data Availability

The data used to support the findings of this study are included within the article.
